The article "The prevalence, perceptions and behaviors associated with traditional/complementary medicine use by breastfeeding women living in Macau: a cross-sectional survey study" was published in 2020. Journal: BMC Complement Med Ther.

# The prevalence, perceptions and behaviors associated with traditional/complementary medicine use by breastfeeding women living in Macau: a cross-sectional survey study

**DOI:** 10.1186/s12906-020-02921-8

**Published:** 2020-04-21

**Authors:** Tingyun Zheng, Weijie Chen, Hao Hu, Yitao Wang, Joanna E. Harnett, Carolina Oi Lam Ung

**Affiliations:** 1 State Key Laboratory of Quality Research in Chinese Medicine, Institute of Chinese Medical Sciences, University of Macau, Macau SAR, China; 2 The University of Sydney School of Pharmacy, The Faculty of Medicine and Health, The University of Sydney, Sydney, Australia

**Keywords:** Breast feeding, Lactation, Traditional medicine, Complementary medicine, Survey, Health personnel, Macau

## Abstract

**Background:**

There is a long history of traditional/complementary medicine (T/CM) use by women during lactation. While it is important to evaluate such use within a scientific paradigm to ensure efficacy and safety, knowledge about the prevalence and characteristics of T/CM use during lactation is limited. This study aimed to generate preliminary data on the prevalence, perceptions and behaviors related to T/CM use by women living in Macau during lactation.

**Methods:**

Between April to June 2018, women aged 18 years or above who had breastfed within the previous 12 months were invited to complete a questionnaire which asked about their perceptions and behaviors related to the use of T/CM while breastfeeding. Chi-square analysis and logistic regressions were used to conduct data analysis.

**Results:**

A total of 500 women completed the survey with 62.6% (95% CI 58.37–66.83) reporting use of at least 1 T/CM while breastfeeding. Of these 48.9% (95% CI 44.67 to 53.13) believed T/CM were safe to take during lactation and 55.6% (95% CI 51.37 to 59.83) suggested there were inadequate resources to assist making an informed decision. Working status, monthly family income and the presence of a breastfeeding-related health problems were associated with T/CM use (all *p* < 0.05). The most commonly used T/CM were *Tetrapanax papyriferus*, lecithin, *Vaccaria segetalis*, docosahexaenoic acid and *Trigonella foenum-graecum* commonly referred to as Fenugreek. The most common reasons for using T/CM were “to unblock milk ducts”, “to increase milk supply” and “to improve baby development”. Women were recommended to use T/CM from multiple sources; 15.0% from health personnel (HP) only, 40.0% received recommendations from non-HP only; and 42.2% from both.

**Conclusions:**

The use of T/CM by women during lactation is common in Macau. The current support and resources available to women during the breastfeeding period to make informed decisions about T/CM use is not standardized nor integrated. The gaps identified in this study provide an opportunity to develop resources and a more defined role for HPs to ensure the appropriate and safe use of T/CM in this population.

## Background

According to the World Health Organization, Traditional Medicine (TM) is the sum total of the knowledge, skills, and practices based on the theories, beliefs, and experiences indigenous to different cultures used in the maintenance of health and management of diseases; and Complementary Medicine (CM) refers to the health care practices that are not part of that country’s own tradition and are not integrated into the dominant health care system [1]. The term Traditional and Complementary Medicine merges the terms TM and CM and encompasses products, practices and practitioners according to the World Health Organization [2]. For the purpose of this study, traditional or complementary medicines (known as “T/CM” hereafter) refers to herbal and related products only which encompasses preparations such as dietary supplements, herbal products, and health supplements but does not include vitamins nor minerals.

There is a long history of T/CM use by women during lactation [3]. A systematic review reported that many women consumed herbal products from different sources during breastfeeding for a wide variety of purposes [4]. However, the efficacy and safety of commonly used herbs remained uncertain. This is mainly because many studies on safety or efficacy of T/CM were of poor methodological quality [4] and regulatory standards regarding market entry of these products vary greatly from one country to another [5]. While traditional evidence is a ‘time honored’ system of handing down knowledge and practices, there remains a need to further evaluate this knowledge and experience within a scientific paradigm to establish both efficacy and safety data [6]. In an era where there is a high prevalence of T/CM use across the world, access to such information is particularly important for special populations including women who are lactating [7–9]. In particular, although there were case reports about adverse effects of T/CM consumed by the mothers on their breastfed infants such as lethargy, hyponia and emesis [10], literature describing and evaluating these effects is scarce [11]. Ensuring breastfeeding women are well informed about the potential benefits and the possible risks associated with the use of T/CM is vital for the well-being of the mothers and their breastfed children. However, a general lack of awareness about the potential risks of the T/CM has been reported [12]. Furthermore, little is known about any safety issues for breastfed children associated with T/CM exposure through breastmilk [13, 14].

To be able to help breastfeeding women make informed choices about the use of T/CM is complex. Consideration needs to be given to the use characteristics of T/CM and the breastfeeding women’s perception of and expectations for such products. However, knowledge about the prevalence and characteristics of T/CM use during lactation is limited. A recent review revealed that since 1995, there were only 9 publications focused on the use of T/CM products during lactation compared to 19 publications related to T/CM use during pregnancy and other childbearing stages [15]. The limited literature about the use of T/CM by breastfeeding women were mostly conducted in western countries including Italy [16], Australia [7] and the USA [12]. The importance of cultural influences and T/CM use has become evident [17, 18]. Therefore, it is important to explore and consider differences in the prevalence and characteristics of T/CM use among a variety of cultures that use T/CM including Asian countries [7, 8, 15, 19, 20].

Therefore, the objective of this study was to investigate the prevalence, perceptions and behaviors related to T/CM use by women living in Macau during lactation. It is expected, that the results of this study can be used to inform developments in research, education and policy that guides the appropriate and safe use of T/CM by women during lactation.

## Methods

### Research design

A cross-sectional survey method was applied in this study.

### Development of questionnaire

The self-administered structured questionnaire used in this study was written in English and Chinese. It was validated through two pilot studies which followed the concepts described by Leavy [21]. The first draft of questionnaire was prepared in English and was informed by (1) the research team’s previous study findings [22–27], (2) other similar studies in the literature on related topics [8, 28–32], (3) consultation with pharmacist and lactation consultant, (4) an online discussion among breastfeeding mothers in the online chat groups, and (5) interviews with two mothers who had used T/CM during breastfeeding. The questionnaire was then translated into Chinese. The questionnaire was first pilot-tested for assessing content validity by a group of 4 health personnel (HP) including 1 physician, 1 pharmacist and 2 nurses; and 1 lactation consultant. All comments were taken into consideration and the questionnaire was amended accordingly. The revised questionnaires were peer-reviewed by 2 other researchers (COLU, JH) in the research team for comprehension and further revisions were made. The questionnaires were then pilot-tested for the second time by 3 breastfeeding mothers who were fluent in both languages to further assess content validity, content consistency comprehension, defective questions and the time needed to complete. Suggested changes were incorporated into the final bilingual questionnaire prior to dissemination.

The questionnaire comprised of 3 sections to address the aims of this study. Section A included questions relating to participant demographics; section B and C collected information about participants’ perceptions and behaviors related to T/CM use respectively.

### Sampling

Data was collected using an online survey targeting women residing in Macau who were 18 years or older, and who was breastfeeding or had breastfed in the previous 12 months.

An estimated sample size based on 6529 live births in 2017 was made [33]. Considering the breastfeeding rate of 88% reported by the Health Bureau [34], the maximum number of breastfeeding women was estimated at 5745 (6529 × 88%). A sample size of at least 361 respondents would provide a target 5% margin of error for population percentage estimates with a level of 95% confidence. Assuming a response rate of 30% based on a previously used recruitment strategy by the authors, a randomized sample of 1204 breastfeeding women would be needed.

### Data collection

In order to minimize selection bias and obtain sufficient responses, multiple avenues were attempted to recruit a diverse range of participant characteristics: breastfeeding mother-to-support groups, community pharmacies and newborn baby supplies retail stores.

Invitations were originally sent to the two government-approved breastfeeding mother-to-support groups in Macau to seek their support with questionnaire dissemination. One of them replied with a positive response. On average, this support group recruited around 1200 new mothers every year and had accumulated over 8000 members since its founding in 2012. The link to the online survey was provided to the person-in-charge of the organization who then disseminated the link to the members through their internal contact. Two follow-up reminders were made by the organization to all members at two weekly intervals. Researchers did not have contact with the members regarding the survey study to minimize any selection bias, and no incentive was provided to participants.

Out of the 300 licensed pharmacies, 30 were selected randomly. Invitations were sent to the mailing addresses obtained from the government official website. The person in-charge were requested to show the link to the online questionnaire to any women who visited their shops and whom they believed might be eligible for the study.

Likewise, two of the newborn baby supplies retail stores were also invited to support this study by distributing the link of the online questionnaire to their customers believed to be eligible. Advertising in social media was also used to advertise the study to the potential respondents.

Data was collected in Macau between April and June 2018. The online questionnaire was hosted by the online questionnaire distribution company Survey Monkey.

### Data analysis

The survey responses were analyzed by using the Statistical Package for Social Sciences (SPSS) version 24 software for Windows. All the data was entered into SPSS, checked by two investigators (TYZ and WJC), and confirmed by two other investigations (HH, COLU). The demographic data of the respondents was analyzed using descriptive statistics. Descriptive statistic and tests of association and predictors (Chi-square analysis and logistic regressions) were used to analyze the demographic data in section A and the perception and behavior data in section B respectively. Alpha was set at 0.05. Whenever the *P*-value was found to be smaller than 0.05, the association would be considered statistically significant at a confidence level of 95%.

### Patient and public involvement

This study aimed to investigate the prevalence, perceptions and behaviors related to T/CM use by breastfeeding women living in Macau. Apart from being the target population of this study, breastfeeding women were consulted during questionnaire design, and asked to assess the time required to complete the questionnaire. It was anticipated that increased awareness about the safe and appropriate use of T/CM would be raised among breastfeeding women by completing and/or knowing about the survey.

## Results

A total of 780 attempts to finish the questionnaire were recorded, in which a total of 500 surveys were completed (completion rate 64%) and no double entry was noted. The sample size resulted in a 4.19% margin of error for population percentage estimates with 95% level of confidence.

### Characteristics of respondents

As presented in Table 1, the majority of the breastfeeding women who completed the survey were over 30 years of age (*n* = 330, 66%), had a university degree (*n* = 435, 87%), and were working (*n* = 426, 85.2%). At the time of the survey study, 181 respondents were still breastfeeding and therefore did not have a definitive period of breastfeeding. For the remaining 319 respondents, 135 or 42% breastfed for more than 12 months. At least 4 out of 5 breastfeeding women reported a breastfeeding-related health condition with ‘blocked milk duct’ (*n* = 311, 62.2%) being the most common complaint. Other common non-specific conditions included general fatigue (*n* = 323, 64.6%) and sleeping problems (*n* = 321, 64.2%). About 38.2% (*n* = 191) also mentioned the experiences of depressive mood.

**Table 1:** Demographic information (*N* = 500) and the factors affecting T/CM use

Demographic information	Number of respondents	Number of users (%)	***P*** Chi-square test
**Total number of participants**	500	313 (62.60)	
**Age**			0.33
≤ 25	13	5 (38.46)	
26 to 30	157	95 (60.51)	
31 to 35	242	154 (63.64)	
36 to 40	78	53 (67.95)	
≥ 41	10	6 (60.00)	
**Cultural background**			0.10
Asian	470	290 (61.70)	
Non-Asian	30	23 (76.67)	
**Marital status**			0.82
Married	480	300 (62.50)	
Not married (Cohabitant, single, Widowed or divorced)	20	13 (65.00)	
**Education**			0.07
Secondary education	65	33 (50.77)	
Higher education	427	276 (64.64)	
Others	8	4 (50.00)	
**Working status**			***0.03***
Working	426	275 (64.55)	
Not working	74	38 (51.35)	
**Average family income every month**^**a**^			***0.04***
< MOP20,000	40	17 (42.50)	
MOP 20,000 - 40,000	115	69 (60.00)	
MOP 40,001 - 60,000	171	108 (63.16)	
MOP 60,001 - 80,000	116	77 (66.38)	
> MOP 80,000	58	42 (72.41)	
**Number of children**			0.86
1	279	176 (63.08)	
2	195	122 (62.56)	
3 or more	26	15 (57.69)	
**The duration of breastfeeding*(N = 319)***^**b**^			0.41
< 1 month	35	20 (57.14)	
1 month - 6 months	82	50 (60.98)	
6 months −12 months	67	42 (62.69)	
> 12 months	135	70 (52.59)	
**Breastfeeding two or more children at the same time**			0.10
No	427	261 (61.12)	
Yes	73	52 (71.23)	
**Suffered from chronic diseases when breastfeeding**			0.07
No	475	293 (61.68)	
Yes	25	20 (80.00)	
**Any breastfeeding-related health conditions when breastfeeding**			***0.00***
No	97	41 (42.27)	
Yes	403	272 (67.49)	

^a^MOP refers to the currency used in Macau (USD 1 is equal to MOP 8 approximately)

^b^181 respondents were still breastfeeding and therefore were not able to answer this question

### Prevalence of T/CM use

Breastfeeding women who used any kind of T/CM to achieve any health benefits for themselves and/or their breastfed children were classified as “users”. Among the 500 respondent, 313 or 62.6% (95% CI 58.37–66.83) indicated that they had used at least 1 T/CM for various beneficial outcomes during lactation. Of these 313 users, 51 (16.3%) reported using only 1 T/CM, 50 (16%) used 2 T/CM, 74 (23.6%) used 3 T/CM, 48 (15.3%) used 4 T/CM, 33 (10.5%) used 5 T/CM, 18 (5.8%) used 6 T/CM, and 39 (12.5%) used 7 or more T/CM. The average number of T/CM used was 4 with a maximum of 17. Duration of use ranged from less than 1 week to more than 6 months. Results of Chi-square test indicated that T/CM use might be associated with the women’s working status (*P* = 0.03), family monthly income (*P* = 0.04), and the presence of breastfeeding-related health problems (*P* = 0.00) (see Table 1).

### Perceptions about the efficacy and safety of T/CM

Two-hundred and forty-five of the breastfeeding women (49%) believed that T/CM were generally safe to take during lactation and 218 (43.6%) were not sure about it (see Fig. 1). When comparing the safety of T/CM to prescription or over-the-counter medicines, 208 (41.6%) agreed that T/CM were safer to take, 205 (41%) were not sure and 87 (17.4%) believed otherwise. Only 46 of the breastfeeding women (9.2%) indicated that there was a sufficient amount of reliable information to inform T/CM use during breastfeeding whereas 278 (55.6%) did not agree so. The majority of them expressed the need for more information about the safety of T/CM to their breastfed children (*n* = 480, 96%), side effects (*n* = 437, 87.4%) and effectiveness (*n*- = 416, 83.2%). Nevertheless, 335 (67%) indicated that they would consider using T/CM during lactation if necessary.

**Fig. 1:** Breastfeeding women’s perception about T/CM

Logistic regression model shows that the use of T/CM during lactation is associated with the positive attitude towards the safety of using T/CM during lactation, and the perceived accessibility of reliable information to inform T/CM use as determined with the above statements with statistic difference (*p* < 0.05) as shown in Table 2.

**Table 2:** Logistic regression model of breastfeeding women’s perception about T/CM and the decision about T/CM use

	Non-users (%)	Users (%)	***p***
***“I think T/CM are generally safe to take during breastfeeding.”***			
Strongly agree/Agree	53/245 (21.6%)	192/245 (78.4%)	***0***
Not sure	112/218 (51.4%)	106/218 (48.6%)	
Strongly disagree/Disagree	22/37 (59.5%)	15/37 (40.5%)	
***“I think T/CM are safer to use while breastfeeding than prescription or over-the-counter medicines.”***			
Strongly agree/Agree	57/208 (27.4%)	151/208 (72.6%)	***0***
Not sure	91/205 (44.4%)	114/205 (55.6%)	
Strongly disagree/Disagree	39/87 (44.8%)	48/87 (55.2%)	
***“I would consider using T/CM during breastfeeding if necessary.”***			
Strongly agree/Agree	65/335 (19.4%)	270/335 (80.6%)	***0***
Not sure	92/126 (73%)	34/126 (27%)	
Strongly disagree/Disagree	30/39 (76.9%)	9/39 (23.1%)	
***“I think there is a sufficient amount of reliable information to inform the use of T/CM during breastfeeding.”***			
Strongly agree/Agree	9/46 (19.6%)	37/46 (80.4%)	***0.009***
Not sure	77/176 (43.8%)	99/176 (56.3%)	
Strongly disagree/Disagree	101/278 (36.3%)	177/278 (63.7%)	

### Users’ choice of T/CM and purposes of T/CM use

Among the 41 T/CM reportedly used by the breastfeeding women, the most commonly used T/CM composed of 5 traditional Chinese medicines and 5 other T/CM: *Tetrapanax papyrifer* (*n* = 242, 77.3%), lecithin (*n* = 223, 71.2%), *Vaccaria segetalis* (*n* = 98, 31.3%), docosahexaenoic acid (DHA) (*n* = 98, 31.3%), *Trigonella foenum-graecum* (*n* = 95, 30.4%), omega-3 fatty acids (fish oil) (*n* = 63, 20.1%), *Fructus hordei germinatus* (*n* = 55, 17.6%), *Sojae semen preparatum* (*n* = 53, 16.9%), *Fructus liquidambaris* (*n* = 53, 16.9%), and *Taraxacum officinale* (*n* = 38, 12.1%) (see Table 3). Around 10% of the users indicated that they did not know what T/CM they took.

**Table 3:** The top ten most common T/CM used by respondents

T/CM	N (% of total users) reported the use	N (% of this user group) indicated this T/CM was effective	Common reasons for use (Number of respondents)								
			Specific to breastfeeding				Non-specific to breastfeeding				
			To unblock milk ducts	To increase milk supply	To reduce milk supply	To relieve breast and nipple pain	To improve the breastfed children’s development	To relieve depressive mood/ stress	To relieve sleeping problems	To improve skin conditions	To enhance energy level
*Tetrapanax papyrifer*	242 (77.3%)	62 (25.6%)	**√** (154)	**√** (83)	**√** (1)	**√** (4)					
Lecithin	223 (71.2%)	54 (24.2%)	**√** (187)	**√** (27)		**√** (7)					
*Vaccaria segetalis garcke*	98 (31.3%)	17 (17.3%)	**√** (26)	**√** (62)	**√** (2)	**√** (1)					**√** (1)
Docosahexaenoic acid	98 (31.3%)	23 (23.5%)		**√** (1)			**√** (75)	**√** (1)		**√** (3)	**√** (2)
*Trigonella foenum-graecum*	95 (30.4%)	19 (20%)	**√** (6)	**√** (84)							
Omega 3 fatty acids (Fish oil)	63 (20.1%)	13 (20.6%)	**√** (4)	**√** (3)			**√** (39)	**√** (1)		**√** (7)	
*Fructus Hordei Germinatus*	55 (17.6%)	6 (10.9%)	**√** (1)	**√** (2)	**√** (50)	**√** (1)					
*Semen Sojae Preparatum*	53 (16.9%)	4 (7.5%)	**√** (1)		**√** (49)				**√**(1)		
*Fructus liquidambaris*	53 (16.9%)	13 (24.5%)	**√** (33)	**√** (12)		**√** (2)			**√** (1)		
*Taraxacum officinale*	38 (12.1%)	9 (23.7%)	**√** (13)	**√** (3)	**√** (2)	**√** (9)	**√** (1)		**√** (2)		**√** (1)

The wide range of reasons for using T/CM can be classified into one of the two groups: specific to breastfeeding, and not specific to breastfeeding (see Table 3). Regarding breastfeeding-specific reasons, T/CM were mostly used to “to unblock milk ducts”, “to increase milk supply”. “to reduce milk supply”, and “to manage breast/nipple pain”. T/CM were also used for health benefits not specifically related to breastfeeding such as “to enhance the development of the breastfed children”, “to relieve depressive mood”, “to relieve sleeping problems”, “to improve skin conditions” and “to enhance energy level”. When asked if they found T/CM effective, only 92 out of the 313 users (29.4%) clearly indicated that the T/CM they used were effective for their purposes of use. The users were also asked about the experiences of adverse effects associated with the use of T/CM and 49 (15.7%) reported having such experiences when they used T/CM during breastfeeding.

### Breastfeeding wosmen’s use of resources to make a decision about T/CM use

Among the users, other than 9 (2.9%) of them who did not receive any recommendations, the majority of users received recommendations from an average of 3.2 sources (range from 1 to 10); 125 (40.0%) from non-HP only, 47 (15.0%) from HP only and 132 (42.2%) from both. As shown in Fig. 2, among the non-HP, 126 users received recommendations about T/CM use from friends, 123 users were recommended by family and relatives, 117 users by social media, 107 users learnt about T/CM from the internet. Eighty-one users learnt about T/CM from breastfeeding social support groups. Other non-HP who might make such recommendations included breast masseuses, confinement lady, and lactation consultants. Among the 5 regulated HP, 165 users were recommended by Chinese Medicine doctors to use T/CM, a much smaller number of users received such recommendations from Western Medicine doctors, physiotherapists, nurses and pharmacists.

**Fig. 2:** Users’ sources of recommendation about T/CM use during breastfeeding

## Discussion

The data collected in this study suggests that over half of adult women residing in Macau use at least one T/CM while breastfeeding despite being unsure about the efficacy and safety of the products, and their decision to use T/CM is informed by both formal and informal sources.

In this study, it was found that over 50% of the women in Macau used at least 1 T/CM during breastfeeding. The findings about the common use of T/CM during breastfeeding are in consistence with what have been previously reported in other countries: 16% in the USA [12], 59.9% in Australia [7], 97% in Italy [16], and 45% in China [8]. While the lower prevalence of T/CM use in the USA may be a true representation, it may also be associated with differences in study design. .

The association that T/CM use while breastfeeding was associated with being a working parent, having a higher family income and having a breastfeeding-related health condition is consistent with studies conducted in the USA, the UK and Australia [35–37]. The association between breastfeeding-related discomfort and T/CM use in this study is not a new finding. However, the demographic characteristics identified in this study indicates there are unmet health care needs related to both physical and psychosocial pressures facing breastfeeding women in Macau who need, or choose to be in the paid workforce.

Our findings that 4 out of 5 women experience lactation related health issues are consistent with other reports. However, women are generally surprised by the extent, intensity and duration of discomfort and pain associated with such conditions [38]. In order to manage these health-related challenges, T/CM use has become a common part of self-care, and self-prescribing with T/CM has been observed in breastfeeding populations all over the world [15]. Therefore, the results of this study and the findings of others suggest there is a need to educate, prepare and support mothers during the entire pre- and antenatal period in managing the physical and emotional challenges they face while breastfeeding [39, 40].

Consistent with previous reports, the use of T/CM in this study was associated with personal preference and a perception that such products are natural, safer and with fewer side effects than conventional treatments [13, 28, 41, 42]. Interestingly, in this study the number of women who perceived T/CM to be safe was substantially lower than those who reported using T/CM during lactation. In other words, some breastfeeding women would choose to use T/CM even when they were unsure about the safety. The lack of cautionary behaviors related to T/CM safety and potential risks associated with T/CM use during breastfeeding warrants attention.

It is important for the T/CM users, especially breastfeeding women, to acknowledge that uncertainties remain regarding the quality, safety, potential herb-herb/conventional medication/disease interactions, and efficacy [43–45]. Whether the T/CM is able to meet certain health claims made on the labels or as advertised is also questionable [43]. An overall lack of standardized regulation of the T/CM and related dietary supplements in most jurisdictions throughout Asia poses further challenges associated with quality assurance and safety monitoring [44]. For instance, in Macau, there is a fine line between the definitions of medicine and non-medicine, which make them subject to regulation of various extent. A product having the same formulation as a medicine may be classified as a non-medicine if certain health claims are removed from the product label [46]. In addition, certain over the counter T/CM may be contaminated by prohibited substances [32, 47]. Use of T/CM related products are also associated with emergency room visits and in the US, an estimate of 23,000 such cases happen every year [48]. Breastfeeding women should be made aware of the risks and benefits before they can make an informed decision about using T/CM when necessary. Two recent studies involving this population reported breastfeeding mothers may experience adverse reactions ranging in severity from mild to serious, including nausea, vomiting, and decreased glucose levels [28, 49]. More extreme cases such as toxic epidermal necrolysis was linked to the use of *Trigonella foenum-graecum* by a young woman [50] and a precaution is warranted for cross-reaction among *Trigonella foenum-graecum* and chickpeas, peanuts, and other legumes in allergic patients is possible [51].

The finding that women practice polypharmacy related to T/CM while breastfeeding women is also concerning. The risks associated with concurrent use of multiple traditional Chinese medicines and other complementary medicines for long periods i.e. more than 6 months is not fully understood. In addition to unknown risks to the mother, it remains uncertain how much of various T/CM constituents make their way to the breast milk and the effects of this on their breastfed infants’ health.

This study indicates the most common reasons women use T/CM were to “to unblock milk ducts” and “to increase milk supply”. This is consistent with previous reports, that the most common use of herbal medicines in breastfeeding women was to improve milk supply [7, 12, 28] or as a traditional prophylactic for insufficient milk production [43] and engorgement [13]. The breastfeeding women in this study also took T/CM, but to a lesser extent, for more general ailments such as depressive moods, headaches and sleeping problems, similar to previous findings [13]. Given the prevalence and potential serious consequences of undiagnosed and untreated post-natal depression, such symptoms should be medically assessed [52]. It has been reported that T/CM use has been associated with delaying proper treatment or masking certain symptoms, resulting in both direct and indirect risks or even harm [53]. The effective management of blocked milk ducts is important in the prevention of mastitis further reiterating the need for women to be fully informed about both the nature of the condition and the limitations of any treatments they may use including T/CM.

The need for standardized information related to self-management with T/CM is further highlighted in this study by some women reporting the use of the same T/CM to promote or reduce milk supply during weaning. Adequate dietary intake of the essential fatty acids plays an important role in normal infant development [54]. Therefore, it is reasonable that some women in this study would choose to supplement their diet with omega 3 fatty acids such as DHA. However, this decision is not fully supported by the results of a large meta-analysis involving 143 studies where the effects of supplementing pregnant or breastfeeding women and infant formulas with omega-3 supplements was assessed [55]. Although a modest increase in the length of gestation and infant birth weight was identified, the overall risk of a low birth weight or premature birth was not. In regards to infants health, omega-3 supplementation were not found to have any effects on the long-term development including growth after birth, visual acuity, long-term neurological and cognitive development, and the risks of autism, and learning disorders [55]. There is also insufficient evidence to support the efficacy of lecithin to unblock milk ducts, increase milk supply and manage breast/nipple pain [56].

Reliable and reputable T/CM information sources are essential to make informed decisions about self-management in health [57]. A women’s health literacy influences her decision about T/CM use during lactation and that decision making process is informed by a web of complexity and multiple information sources [19]. Our findings are similar to other studies, with breastfeeding women reporting a diverse social network and the source of information about T/CM was mainly from friends/family and the media, while HPs such as physicians and nurses only played a small part in providing T/CM-related information [7, 58]. The reliability and accuracy of information originating from anecdotal reports within a women’s social network may not always be reliable [19, 58]. Furthermore, T/CM product promoting websites can also be a potential source of misinformation [59].

The interesting finding in this study is that nearly half of women consulted both social and professional sources of information thus raising a real opportunity for HPs to play a role. Given the demographic region of this study, it was not surprising that TCM doctors were acknowledged as a trusted information source and confirms previous reports [60]. The finding that other HPs had little to no role in advising about T/CM is in keeping with a European study which revealed that the role of physicians as sources of T/CM information was low [58]. Only 18.6% actually providing information to patients and the number was even lower among nurses with only 3% of nurses were identified as the main source of information for patients in that study [58]. It is also important to note that the lack of participation of pharmacists in the decision-making process about T/CM use among the breastfeeding women identified in this study contradicts many breastfeeding women’s expectations. In a recent literature review about the role HP in advising breastfeeding women about T/CM use, 17 out of the 22 included studies either discussed about or specifically focused on the role pharmacists can play in helping breastfeeding women make informed decision about T/CM use [25]. As medicines experts, pharmacists are considered a reliable information source by breastfeeding women [25, 61]. The significant gaps in the support breastfeeding women received from HPs about their use of T/CM raises an argument raised by women that all HPs should be knowledgeable of benefits and risks of T/CM [12, 13, 50, 61, 62].

Other than TCM doctors, another major contributor of T/CM information were breastfeeding consultants. Although not regulated as a HP in Macau, some breastfeeding consultants such as International Board Certified Lactation Consultants are trained to provide support in the overall management of breastfeeding and their role as a trustworthy provider of care in promoting breastfeeding is well established [63, 64]. This opens a potential opportunity to be a reliable source of T/CM information. Clearly, standardized peer reviewed information and guidelines for breastfeeding women and those that care for them are needed [16, 62, 65–67].

### Strengths of this paper

The study is the first study to be conducted in Macau on this topic. Macau is a unique representation of the Asia region where both traditional Chinese and western medicine are commonly used, either alone or in a concurrent manner. Our recruitment procedure provides a broad representation of eligible women through access to breastfeeding mothers groups, community pharmacies and retail outlets.

### Limitations

A limitation often associated with the type of data collected in this study relates to the reliance on self-reporting by participants. Self-reporting is associated with an increased risk of responder and recall bias. The survey instrument was designed for a simple descriptive scoping study and as such the scales developed have not been tested and validated.

## Conclusions

The use of T/CM by women during lactation is common in Macau. The current support and resources available to women during the breastfeeding period to make informed decisions about T/CM use is not standardized nor integrated. The gaps identified in this study provide an opportunity to develop resources and a more defined role for HPs to ensure the appropriate and safe use of T/CM for women and their breastfed infants.

## Data Availability

The datasets used and/or analysed during the current study are available from the corresponding author on reasonable request.

## Abbreviations

T/CM: Traditional/complementary medicine
HP: Health personnel
SPSS: Statistical Package for Social Sciences
